RETRACTED

# Reversal Effect of ST6GAL 1 on Multidrug Resistance in Human Leukemia by Regulating the PI3K/Akt Pathway and the Expression of P-gp and MRP1

**DOI:** 10.1371/journal.pone.0085113

**Published:** 2014-01-16

**Authors:** Hongye Ma, Lei Cheng, Keji Hao, Yanping Li, Xiaobo Song, Huimin Zhou, Li Jia

**Affiliations:** 1 College of Laboratory Medicine, Medical University, Dalian, Liaoning Province, China; 2 Department of Laparoscopic Surgery, the First Affiliated Hospital of Dalian Medical University, Dalian, Liaoning Province, China; 3 Department of Nuclear Medicine, People's Hospital of Peking University, Beijing, China; 4 Department of Medical Biology, Faculty of Health Sciences, University of Tromsø, Tromsø, Norway; 5 Department of Microbiology, Dalian Medical University, Dalian, Liaoning Province, China; Wayne State University, United States of America

## Abstract

β-galactoside α2, 6-sialyltransferse gene (ST6GAL) family has two members, which encode corresponding enzymes ST6Gal I and ST6Gal II. The present atudy was to investigate whether and how ST6GAL family involved in multidrug resistance (MDR) in human leukemia cell lines and bone marrow mononuclear cells (BMMC) of leukemia patients. Real-time PCR showed a high expression level of ST6GAL1 gene in both MDR cells and BMMCs (*P<0.05). Alternation of ST6GAL1 levels had a significant impact on drug-resistant phenotype changing of K562 and K562/ADR cells both in vitro and in vivo. However, no significant changes were observed of ST6GAL2 gene. Further data revealed that manipulation of ST6GAL1 modulated the activity of phosphoinositide 3 kinase (PI3K)/Akt signaling and consequently regulated the expression of P-glycoprotein (P-gp, *P<0.05) and multidrug resistance related protein 1 (MRP1, *P<0.05), which are both known to be associated with MDR. Therefore we postulate that ST6GAL1 is responsible for the development of MDR in human leukemia cells probably through medicating the activity of PI3K/Akt signaling and the expression of P-gp and MRP1.

## Introduction

MDR and disease relapse are often regarded as the causes of the failure of chemotherapeutic drug treatments in patients diagnosed with malignant neoplasm including leukemia [1]. Numerous reports have focused on the mechanisms of MDR of tumor cells, for example the expression of drug transporting pumps, changes in the targets of anticancer drugs, decrease of drug activity, as well as changes in apoptosis regulatory pathways that contribute to MDR [2]–[4]. MDR is conventionally regarded as the consequence of overexpression of transporter proteins belonging to the ATP binding cassette (ABC) family such as P-gp and MRP1, which lead to lower intracellular drug accumulation and hence reduce cellular toxicity of chemotherapeutic agents [5]. Recently, researchers pay more attention to the relationship between glycan alterations and resistance to chemotherapy of neoplastic cells. Although structure modifications of glycans have been observed in drug-resistance leukemia cells, little is known about the effects of glycosyltransferases or relevant glycogenes on the development of leukemia drug-resistance [6], [7].

RETRACTED

Sialic acids, which are terminal monosaccharide attached to glycan chains of cell surface, are commonly found in glycoconjugates. Various sialic acid decorations on the cell surface are shown to be involved in many biological processes, such as cell recognition, cell adhesion, receptor activation, cancer progression, metastatic spread and signal transduction [8]–[9]. ST6GalI is a sialyltransferase that links the sialic acid residues to terminal galactose of glycan chains by α- 2, 6-linkage [10]. It distributes widespread tissue-specific distribution in mammals, and the aberrant expression of ST6GalI is often related to poor prognoses in colon, epithelial tumors, gastric cancers and acute myeloid leukemia [6], [11]–[13]. Overexpression of ST6GalI was involved in chemotherapy resistance in ovarian tumor cells [14]. The altered levels of ST6GalI were also found in Hca-F and Hca-P murine hepatocarcinoma cells with differed invasive properties both *in vitro* and *in vivo* [15]. In contrast to ST6GalI, ST6GalII, a recently identified additional sialyltransferase, confines to human intestine, colon and brain [16], [17]. It exhibits relatively low and no activities toward some glycoproteins and glycolipids respectively and seems to recognize oligosaccharides to glycoproteins as acceptor substrates [18], [19]. Tremendous studies have focused on the involvement of sialylation in tumorigenesis, but the relationship between ST6GalI or ST6GalII and MDR remains unclear.

PI3K/Akt signaling activation might be implicated in the progression of a wide variety of neoplasias [20]. Recent research illustrated that aberrant activation of PI3K/Akt pathway contributed to the survival and drug resistance of different types of human neoplasm cells [21], [22]. Activation of Akt was associated with poor prognosis and chemotherapeutic resistance in pediatric B-precursor acute lymphoblastic leukemia [23]. In leukemic cells, chemoresistance was shown to be maintained by PI3K/Akt signaling activation, and could be reversed by LY294002, a known PI3K/Akt antagonist [24]. PI3K/Akt kinase pathway also modulated P-gp-mediated multidrug resistance in L1210/VCR mouse leukemic cell line [25]. But Tazzari showed that that in human acute myelogenous Leukemia (AML) blasts a strong correlation exists between upregulation of the PI3K/Akt survival pathway and MRP1 expression, whereas such a relationship was not found for the P-gp [26]. However, little is known regarding the effect of the signaling pathways on ST6GalI, ST6GalII-mediated leukemia MDR.

RETRACTED

The aims of the present study were to determine sialylated oligosaccharide alterations and the expression level of ST6GAL family among the four pairs of parental and chemoresistant human leukemia cell lines. In addition, we examined the regulation of ST6Gal I or ST6Gal II in leukemia MDR via PI3K/Akt pathway and the possible mechanisms.

## Results

### Differential expression of ST6GAL1, ST6GAL2 in four pairs of leukemia cell lines

To analyze the expression profiles of ST6GAL family in drug sensitive and MDR cells, a real-time RT-PCR analysis was performed. ST6GAL1 was significantly expressed at an elevated level in four MDR cell lines compared with those of four drug-sensitive parental cell lines. By contrast, no significant change of ST6GAL2 was observed. Western blotting analysis further confirmed the enzyme expression in drug sensitive and MDR cells at protein level. These data indicated that differential ST6GAL1 expression might be associated with MDR of leukemia, as illustrated in Fig. 1A and B.

**Figure 1:** Differential expression of ST6GAL1 and ST6GAL2 in four pairs of leukemia cell lines. (A) The mRNA levels of ST6GAL1 and ST6GAL2 analyzed by real-time PCR. Four ADR cells expressed higher levels of ST6GAL1 mRNA than their parental cell types (*P<0.05). No significant changes of ST6GAL2 were observed. (B) Western blotting analysis of ST6GalI and ST6GalII at protein levels. GAPDH served as a control. Data are the means ± SD of triplicate determinants.

### Suppression of ST6GAL1 gene enhances chemosensitivity of K562/ADR cells in vitro and in vivo

Due to the significant increase of ST6GAL1 mRNA and protein expression in K562/ADR cells, we silenced, by shRNA, ST6GAL1 to elucidate the direct implication of ST6GAL1 in the chemosensitivity of K562/ADR cells. As shown in Fig. 2A and B, the expression of ST6GAL1 was significantly reduced in K562/ADR-shRNA transfectants compared with control transfectants both at transcription and protein level. K562/ADR-shRNA-1 transfectant was chosen for the following experiments.

**Figure 2:** Silence of ST6GAL1 gene enhances the chemosensitivity of K562/ADR cell both in vitro and in vivo. (A) ST6GAL1 transcript was decreased apparently in K562/ADR cells by shRNA treatment. (B) After shRNA transfection, distinct reduction of ST6Gal 1 was observed at protein levels by western blotting analysis. (C) Cell chemosensitivity was assessed by cytotoxicity assays. The reported values are the IC_50_ (Mean ± SD) of three independent experiments. IC_50_ represents the drug concentration producing 50% decrease of cell growth. *P<0.05 vs K562/ADR-control shRNA cells. (D) When exposed to adriamycin, the tumor volume of nude mice bearing K562/ADR-ST6GAL1 shRNA-1 xenograft was significantly diminished (*P<0.05). (E) Down-regulation of ST6GAL1 was also shown by IHC staining in xenograft tumors derived from K562/ADR-ST6GAL1 shRNA-1 cells (400×). (F) Flow cytometry analysis showed a lower expression of ST6GAL1 in K562/ADR cells with ST6GAL1 transfection. The data are means ± SD of 3 independent assays (*P<0.05).

RETRACTED

After ST6GAL1 shRNA transfection, the ability of adriamycin, paclitaxel and vincristine to inhibit the growth of K562/ADR was evaluated by MTT assay. The results showed that IC_50_ values were significantly decreased in K562/ADR-ST6GAL1 shRNA group compared to the control, suggesting that cell proliferation was inhibited by therapeutic drug and chemosensitivity was remarkably restored when ST6GAL1 gene was suppressed (Fig. 2C).

To investigate how knockdown of ST6Gal1 gene impacted on chemosensitivity of leukemia cells, we used nude mice bearing K562/ADR and K562/ADR-ST6GAL1 shRNA-1 xenografts to analyze the differences of tumor volumes when therapeutic drugs were administrated. A significant reduction of mean tumor volume of K562/ADR-ST6GAL1 shRNA-1 tumor was observed, as compared with K562/ADR-control shRNA (Fig. 2D). After the measurement of tumor volume, tumors were sectioned for IHC staining analysis of ST6GalI expression pattern, the expression of it was reduced in the mice group with shRNA treatment compared to untreated group or control group (Fig. 2E).

In addition, α-2, 6 sialylation level at the cell surface, detected by FITC-conjugated SNA, was also decreased by treatment with shRNA in K562/ADR cells (Fig. 2F).

### Overexpression of ST6GAL1 gene mediates MDR in K562 cells in vitro and in vivo

To explore the effect of ST6GAL1 on chemosensitivity, a K562 cell line stably expressing ST6GAL1 was established. It was found that the levels of ST6GAL1 mRNA, protein and α2, 6-linked sialic acid were increased notably in ST6GAL1 transfectants (Fig. 3A.B.F). The IC_50_ values for the drugs were significantly increased in the K562/ST6GAL1 group than those in the K562/mock group. Thus, the overexpression of ST6GAL1 in K562 cells resulted in decreased chemosensitivity to antitumor drugs in vitro (Fig. 3C).

**Figure 3:** Overexpression of ST6GAL1 gene enhances the chemoresistance of K562 cells both in vitro and in vivo. After transfection, ST6GAL1 mRNA (A) and protein (B) were increased notably in K562 cells by real time PCR and western blot. (C) Cell chemosensitivity was assessed by cytotoxicity assays. The reported values are the IC_50_ (Mean ± SD) of three independent experiments. IC_50_ represents the drug concentration producing 50% decrease of cell growth. *P<0.05 vs K562/mock cells. (D) An increase of mean tumor in mice group with K562/ST6GAL1 was observed, as compared with that in K562 group and K562/mock group. Within K562/ST6GAL1 group, an increase of tumor growth was found in group without ADR, compared with that with ADR (*P<0.05). (E) Up-regulation of ST6GAL1 was also shown by IHC staining in xenograft tumors derived from K562/ST6GAL1 cells (400×). (F) Increased expression of ST6GAL1 was detected by flow cytometry analysis in K562/ST6GAL1 cells. The data are means ± SD of 3 independent assays (*P<0.05).

RETRACTED

Nude mice were inoculated with tumor cells K562, K562/mock and K562/ST6GAL1. Tumor volumes were measured and compared between the groups with or without adriamycin treatment. Fig. 3D showed that in the group of mice bearing K562 tumors, tumor volumes with adriamycin treatment were lower than those without. But in the group of mice bearing K562/ST6GAL1 tumors, tumor volumes increased significantly even after adriamycin treatment. High expression level of ST6GalI in tumor cells of K562/ST6GAL1 was also validated by IHC staining, as shown in Fig. 3E. Thus, overexpression of ST6GAL1 gene in K562 cells led to raised resistance to chemotherapy.

### Effect of ST6GAL1-activated PI3K/Akt signaling pathway on the expression of P-gp and MRP1 expression

It has been reported that the PI3K/Akt signaling pathway is activated in K562 cell line [27]. Here, we assessed the activity of the PI3K/Akt signaling by ST6GAL1 shRNA-1 treatment in K562/ADR cells. Western blotting (Fig. 4A) showed that the levels of P110α (the catalytic subunit of PI3K), phosphorylation of Akt at Ser473 and Thr308, and NF-κB were significantly reduced with shRNA transfection. However, there was no change in the total amount of Akt protein. Conversely, over-expression of ST6GAL1 in K562 cells enhanced proteins expression of P110α, Akt Ser473, Akt Thr308, and NF-κB, as illustrated in Fig. 4B.

**Figure 4:** Effect of ST6GAL1-activated PI3K/Akt signaling pathway on the expression of P-gp and MRP1. (A) The main molecules of PI3K/Akt pathway were repressed at protein levels with ST6GAL1 shRNA transfection in K562/ADR cells. (B) The increased protein levels of PI3K/Akt signaling molecules were determined by western blot in K562/ST6GAL1 cells. (C) Decreased expression of P-gp and MRP1 were examined by flow cytometry analysis in K562/ADR-ST6GAL1 shRNA cells. (D) Flow cytometry analysis revealed a higher co-expression of P-gp and MRP1 in K562 cells with ST6GAL1 transfection. The data are means ± SD of 3 independent assays (*P<0.05).

RETRACTED

P-gp and MRP1 are the recognized molecules which contributed to the development of MDR [5]. Hence, we investigated whether ST6GAL1 could influence the expression of P-gp and MRP1. Interestingly, flow-cytometric analysis (Fig. 4C and 4D) illustrated that elevated expression levels of P-gp and MRP1 were detected in K562/ST6GAL1 cells compared to those of control cell groups. In addition, K562/ADR cells expressed lower levels of P-gp and MRP1 with ST6GAL1 supression. Therefore, the data might indicate an additional mechanism of ST6GAL1 in MDR of leukemia cells.

### Inhibition of PI3K/Akt pathway increases the chemosensitivity of K562/ADR cells both in vitro and in vivo

In order to explore the activity of PI3K/Akt signaling pathway on chemoresistance of K562/ADR cells, PI3K/Akt pathway was pharmacologically inhibited. As seen in Fig. 5A, K562/ADR cells with LY294002 treatment or Akt siRNA showed obviously decreased protein levels of the main signal molecules of PI3K/Akt pathway. By MTT assay *in vitro*, we observed the inhibition of PI3K/Akt pathway sensitized K562/ADR cells to chemotherapy (Fig. 5B), the similar results were also observed by *in vivo* chemosensitivity analysis, reduced tumor volumes were detected in mice group bearing K562/ADR tumors with impaired PI3K/Akt signaling (Fig. 5C). Altered expression levels of the main signal molecules of PI3K/Akt pathway in mice group bearing K562/ADR tumors with LY294002 or Akt siRNA treatment were also validated by IHC staining, as shown in Fig. 5D

**Figure 5:** PI3K/Akt inhibition changes the chemosensitivity of K562/ADR cells both in vitro and in vivo. (A) The K562/ADR cells were pretreated LY294002 or Akt siRNA. Expressions of PI3K/Akt signaling molecules were then examined by western blot analysis. LY294002 or Akt siRNA treatment also alleviated chemoresistance of K562/ADR cells, revealed by *in vitro* (B) and *in vivo* (C). (D) Down-regulation of PI3K/Akt signaling molecules was also shown by IHC staining in xenograft tumors derived from LY294002 or Akt siRNA treatment cells (400×). (E) Flow cytometry analysis showed that inhibition of PI3K/Akt pathway resulted in reduced levels of P-gp and MRP1. The data are means ± SD of 3 independent assays. ^*^P<0.05 vs DMSO treatment cells; ^#^P<0.05 vs control siRNA treatment cells.

Moreover, to investigate whether suppression of PI3K/Akt signaling activity could influence the expression of P-gp and MRP1, a flow-cytometric analysis was carried out. Lower levels of P-gp and MRP1 were present in K562/ADR cells with LY294002 or Akt siRNA treatment (Fig. 5E). The results implicated a role for PI3K/Akt signaling in regulating P-gp and MRP1 expression and modulating the chemoresistance of K562/ADR cells.

RETRACTED

### Overexpression of ST6GAL1 is detected in patients' AML and CML cases with chemoresistance

Expression of MDR-related marker, ST6GAL1 and ST6GAL2 in leukemia patients is summarized in Table 1. The frequency of P-gp positivity was 92.1% (70 of 76) in AML patients and 86.2% (25 of 29) in CML patients. Then patients were divided into four groups: AML without MDR, AML/MDR, CML without MDR and CML/MDR. As was shown in Table 2, there was a significant difference in the expression of ST6GAL1 between AML/MDR patients (91.4%, 64 of 70) and those without MDR (16.6%, 1 of 6). Accordingly, the proportion of ST6GAL1 positive CML/MDR samples was 90.9% (20 of 22), this was found to be significantly higher than the chemosensitive CML group (28.5%, 2 of 7). However, expression of ST6GAL2 showed no difference between drug resistant groups and chemosensitive groups. According to these results, it was further confirmed the role of ST6GAL1 over-expressions in drug resistance of leukemia cells.

**Table 1:** Clinicopathologic characteristics of the leukemia patients.

Patients Demographics	Subcategory	AML(n = 76)			CML(n = 29)
		M2	M3	M5	
Gender	Male	24	19	10	19
	Female	11	8	4	10
Age(years)	Median	42	44	38	53
	Range	15–79	18–70	12–70	17–76
Splenic enlargement		25	18	10	21
Hemoglobin<110.0 g/L		34	25	12	28
WBC count (10^9^/L)	20–100	19	17	7	2
	>100	2	0	1	27
Platelet count (10^9^/L)	<300	32	26	14	20
	>300	3	1	0	9
P-gp (+)		33	24	13	25
MRP1 (+)		31	23	12	26
ST6GAL1(+)		30	22	13	22
ST6GAL2(+)		6	5	3	4

**Table 2:** The differential expression of ST6GAL1 and ST6GAL2 between MDR and chemosensitive patients.

	AML(n = 76)		CML(n = 29)	
Group	MDR	Chemosensitivity	MDR	Chemosensitivity
	70	6	22	7
ST6GAL1(+)	64 (91.4%)*	1 (16.6%)	20 (90.9%)*	2 (28.5%)
ST6GAL2(+)	13 (18.6%)	1 (16.6%)	3 (13.6%)	1 (14.3%)

P<0.05 vs. patients without MDR.

## Discussion

Clinically chemotherapy resistance is the result of interaction of numerous biological variables [28]. MDR, as an issue with increasing concern, contributes to the chemotherapy failure in leukemia. Recently, some progresses have been gained in revealing the mechanism of MDR [29]. Our study continued to investigate the role of ST6GalI in mediating MDR in human leukemia cells and its possible mechanisms.

Aberrant expression of sialylated glycans has been detected in carcinomas of pancreas, gastric, breast, bladder, brain and colon [30]–[34]. In this study, we found the expression profiles of ST6GAL1 in four pairs of human leukemia cell lines and in the tumor cells of leukemia patients by using a real-time PCR analysis. All the leukemia cells with MDR were characterized with higher expression levels of ST6GAL1 compared to the cells without MDR. ST6GAL1 is known to be involved in the process of proliferation, invasion, and apoptosis of cancer cells [35], [36]. From our results we postulate that abnormal expression of ST6GAL1 also involves in the development of MDR possibly, another malignant behavior of tumor cells. There was not a significant difference of ST6GAL2 expression between the cell groups with or without MDR.

RETRACTED

As up-stream regulators of glycoproteins, glycosyltransferases catalyzed the biosynthesis of glycans. They often exhibit abnormal activity in tumors and participate in the process of drug-resistance development [37]. Zhang et al have observed an elevated level of ST6GAL1 in drug resistance cell line K562/ADR [7]. However, a comprehensive understanding of how ST6GAL1 correlated with the MDR of human leukemia cells was not currently available. In this study, we targeted ST6GAL1, which was over-expressed in K562/ADR cells, and altered the expression levels of the glycogene. A link was found between differential expression levels of ST6GAL1 and changed drug-resistant phenotypes of K562 and K562/ADR cells both in vitro and in vivo (Fig. 2, 3). Thus, based on this insight we hypothesized that ST6GAL1 might function as a critical factor involved in MDR.

The PI3K/Akt signal transduction pathway plays a pivotal role in controlling neoplastic cell growth, survival, motility, invasion and drug resistance [38]–[40]. Recent data has confirmed the correlation of the ST6GAL1-mediated PI3K/Akt signaling pathway with multidrug resistance [36], [40]. Increasing evidences showed that PI3K/Akt signaling was frequently activated in AML cell lines and patient blasts and strongly contributed to proliferation, survival, and drug resistance of these cells [41]–[45]. Akt1 activity/phosphorylation was also up-regulated in MDR human T-lymphoblastic leukemic CEM cells [46]. Here, we demonstrated that the K562/ADR cell line presented higher PI3K/Akt activity than the sensitive one, which was in accordance with the MDR phenotype. Altered expression of ST6GAL1 remarkably modulated the activity of PI3K/Akt pathway in human leukemia cell lines. Furthermore, blockage of PI3K/Akt pathway by Akt-specific inhibitor, LY294002, or Akt siRNA reversed ADR cells to chemosensitivity, indicating that ST6GAL1 might promote the development of MDR probably through activating the PI3K/Akt signaling pathway (Fig. 5). Thus, consistent with already reported results, LY294002 can antagonize P-gp-mediated multidrug resistance [25].

RETRACTED

It has been reported that the PI3K/Akt signaling enhances drug efflux by ATP-binding cassette (ABC) transporters in order to maintain MDR of tumor cells [47]. ABC transporters are a superfamily of transmembrane proteins that transports a wide variety of substrates across cell membranes. They are found on the surface of normal cells and various cancer cells, where they play significant roles in the development of MDR [48]. As two main members of ABC transporters, P-gp and MRP1 are frequently used as markers to screen MDR patients clinically. MRP1 expression is also under the control of the PI3K/Akt signal transduction network in human acute myelogenous leukemia blasts [26]. We found a positive relationship between the levels of P-gp and MRP1 and the expression level of ST6GAL1, as well as the activity of PI3K/Akt signaling in K562 and K562/ADR cell lines. Since ST6GAL1 was observed as regulatory gene on the activity of PI3K/Akt signaling, we assumed that ST6GAL1 might increase the expression of P-gp and MRP1 through PI3K/Akt pathway, thereby mediating MDR of leukemia cells.

In summary, our results demonstrate an association between differential expression of ST6GAL1 and changed MDR phenotypes of leukemia cells. The possible mechanism is ST6GAL1 activating the PI3K/Akt signaling pathway that results in the expression of P-gp and MRP1. However, drug resistance is multifactorial event, and multiple glycomic alterations could also be responsible for these phenotypes. Therefore, the molecular machanism of tumor MDR remains to be further investigated.

## Materials and Methods

### Cells

Four human leukemia cell lines, including a chronic myelogenous leukemia cell line (K562), an acute myelogenous leukemia cell line (HL60), an acute promyelocytic leukaemia cell line (NB4), and a leukemic monocytic cell line (U937) were obtained from the KeyGEN Company (China). All cell lines were cultured in RPMI 1640 medium (Gibco, Grand Island, NY, USA) supplemented with 10% heat inactivated fetal bovine serum (Gibco) and 1% penicillin-streptomycin (Gibco) at 37°C in a humidified atmosphere containing 5% CO2. Adriamycin (Sigma) was added to parental cell cultures in stepwise increasing concentrations from 0.1 µg/ml to 5 µg/ml for 2 months to develop an adriamycin-resistant (ADR) subline, namely K562/ADR, HL60/ADR, NB4/ADR and U937/ADR, correspondingly. To maintain the MDR phenotype, the complete medium of the resistant cell clones were supplemented with 1.0 mg/L adriamycin. ADR cells were maintained in complete medium without adriamycin for one week and cells with >90% viability prior to subsequent treatments.

### Samples from leukemia patients

The study cohort was made up of 105 previously untreated leukemia patients, including 76 cases of acute myeloid leukemia (AML) and 29 cases of chronic myeloid leukemia (CML). All patients were obtained in the First Affiliated Hospital of Dalian Medical University between April 2010 and July 2012, and they provided written informed consent, and the institutional ethics committees of the First Affiliated Hospital of Dalian Medical University approved the study as well as contents of the written consent. The leukemic subtypes of AML were determined according to the French-American-British classification as follows: 35, 27 and 14 cases of M2, M3 and M5, respectively. Patients' clinical characteristics were given in Table 1. The diagnosis of AML and CML was based on cytomorphology, cytochemistry, multiparameter flow cytometry, immunology, molecular genetics and cytogenetics.

RETRACTED

### Separation of leukemic blast cell

BMMC were separated by Ficoll-Hypaque density gradient centrifugation from bone marrow or peripheral blood taken at the initial diagnosis and were cultured in plastic dishes to remove adherent cells at 37°C for 24 h. Freshly separated non-adherent cells were maintained in modified Dulbecco's medium containing 10% fetal bovine serum, 10 mM β-mercaptoethanol, 2 mM L-glutamine, 50 ng/mL human stem cell factor, 10 ng/mL human interleukin-3, and 10 ng/mL human interleukin-6. The expressions of P-gp and MRP1 were measured by flow cytometric assays to determine the resistant phenotype of patients. ST6GAL1 and ST6GAL2 levels of all patients were determined by real time PCR.

### Real Time PCR analysis

Total RNA was isolated with Trizol reagents (Gibco BRL, Rockville, MD, USA) and cDNA was synthesized using QuantiTect Reverse Transcription Kit (QIAGEN, valencia, CA) according to the manufacturer's protocol. Real time PCR was carried out on a Roche LightCycler480 real time PCR system (Applied Biosystems, Foster City, CA) using QuantiTect SYBR Green PCR Kit (QIAGEN, valencia, CA). After a denaturation and polymerase activation step (15 min at 95°C), 40 cycles of denaturation (15 s at 94°C), annealing (30 s at 58°C) and extension (30 s at 72°C) were run. The sequences of the primers used for the real-time PCR assays were as follows: 5′-CTTGTTTTCCTGCTCAGA-3′ and 5′-GCAAACAGAAGAAAGACCA- 3′ for ST6GAL1, 5′-ACGCTGCTGATTGACTCTTCT-3′ and 5′-CACATACTGGCA CTCATCTAA-3′ for ST6GAL2; 5′-CTCCTCCACCTTTGACG-3′ and 5′-CACCACC CTGTTGCTGTA-3′ for GAPDH, the expression of target gene was determined relative to GAPDH and calculated as 2^−(Ct^_Target gene_^−Ct^_GAPDH_^)^.

### Western blot analysis

Total cell protein were electrophoresed in 10% SDS-PAGE gel and blotted onto a polyvinylidene difluoride membrane. After being blocked with 5% powdered skim milk for 2 h in phosphate-buffered saline containing 0.1% Tween 20 (PBST), the membranes were incubated with antibody (1∶500 diluted, Abcam, Cambridge, UK), overnight at 4°C, and then incubated with secondary antibody anti-rabbit/mouse-HRP (1∶2000 diluted, Santa Cruz Biotech, Santa Cruz, CA). GAPDH antibody (1∶200 diluted, Santa Cruz Biotech, Santa Cruz, CA) was used as a control. All bands were detected using ECL Western blotting kit (Amersham Biosciences, UK), according to the manufacturer's instruction.

RETRACTED

### Deregulation of ST6GAL1 in K562/ADR cells by RNAi

K562/ADR cells were transferred to a 6 well plate which was seeded 5×10^5^ cells in 1 ml of growth medium in each well and incubated at 37°C in a CO_2_ incubator. The cell cultures were transfected with ST6GAL1 shRNA-1, ST6GAL1 shRNA-2 and ST6GAL1 shRNA-3 (Thermo Fisher, Inc, 178042). Scrambled shRNA was used as the negative control. ST6GAL1 shRNAs were mixed with Lipofectamine™ 2000 (Invitrogen). Transfer cells were cultured and incubated at 37°C for 6 h, followed by incubation with complete medium for additional 24 h. Then cells were harvested for further study. The cell transfection efficiency was 85% by fluorescent microscope and the cell viability was 90% by trypan blue dye exclusion assay.

### Over-expression of ST6GAL1 in K562 cells

The human ST6GAL1 coding region were obtained from TaKaRa company (Dalian, China) and were inserted into the pEGFP-N1 vector (Invitrogen, Carlsbad, CA) respectively using EcoRI, XhoI sites. Cells were transfected with 5 µg of target gene expression vector or empty vector (EV) in 100-mm dishes using TurboFect Transfection Reagent (QIAGEN, valencia, CA) according to the manufacturer's instruction. After 60 days of screening, the cell lines stably expressing ST6GAL1 (K562/ST6GAL1), and empty vector (K562/mock) were established. Then cells were collected for further explorations.

### In vitro drug cytotoxic assay

MTT assay was used to measure the drug resistance. 1×10^4^ cells per well were plated in 96-well plate and incubated with different anticancer drugs paclitaxel, vincristine, and adriamycin (Sigma, St. Louis, MO) for 48 h, respectively. Then cells were treated with 100 µl MTT (0.5 mg/ml, Sigma). After 4 h incubation at 37°C in 5% CO_2_, 100 µl DMSO (Gibco) was pipetted to solubilize the formazan product for 30 min at room temperature. The spectrometric absorbance was measured at 490 nm by microplate reader (Model 680; Bio-Rad, Hercules, CA). Each test was repeated three times. The drug resistance was estimated by comparing the IC_50_ values (drug concentration that inhibits cell growth by 50%) from growth inhibition curves.

RETRACTED

### In vivo chemosensitivity assay

Five-week-old nude mice were obtained from Animal Facility of Dalian Medical University and were provided with sterilized food and water. Approximately, 1×10^7^ K562 and 1×10^7^ K562/ADR viable cells were injected subcutaneously into the right flank of each nude mouse. When mice bearing palpable tumors (about 1 week after tumor cell inoculation), K562, K562/ST6GAL1, K562/mock, K562/ADR, K562/ADR-control shRNA, K562/ADR-ST6GAL1 shRNA-1 tumor-bearing mice were randomly divided into control and treatment groups (n = 6 animals per group). The treatment groups received 7 mg/kg adriamycin i.p. three times a week for 3 weeks, and the control groups received physiological saline alone. Mice were sacrificed and their tumors were isolated, weighed, and photographed. The tumor volume was calculated by the following formula: Tumor volume = 1/2(length×width^2^). Experiments were approved by the Committee on the Ethics of Animal Experiments of the Dalian Medical University, China (Permit Number: 12-896).

### Immunohistochemical (IHC) staining analysis

Visible tumors were removed from the mice and immunohistochemistry was performed on paraffin embedded sections. The slides were dried, deparaffinized, rehydrated. After deparaffinization and blocking of endogenous peroxidase, the slides were labeled overnight at 4°C with antibodies (Abcam, Cambridge, UK) at a dilution of 1∶200. The following staining was performed at room temperature for 60 min with secondary streptavidin-HRP-conjugated antibody (Santa Cruz Biotech, Santa Cruz, CA). Finally, the sections were counterstained with hematoxylin and cover-slipped. The Image-Pro Plus4.5 Software (Media Cybernetics, USA) was used to analyze the expression of proteins.

### Inhibition of the PI3K/Akt signaling

LY294002 (Sigma) or Akt siRNA was used to suppress the activity of the PI3K/Akt signaling in K562/ADR cells. Briefly, cells (1×10^4^ cells per well) were incubated with dimethyl sulfoxide (DMSO), the PI3K inhibitor LY294002 (10 µM) dissolved in DMSO, Akt control siRNA and Akt siRNA. Cells were collected after 24 h. Changes in chemosensitivity and gene expression were measured by MTT assay and western blot analysis, respectively. Each experiment was run in triplicate to determine means and SDs.

### Flow cytometry analysis

Tumor cells were washed with 1×phosphate buffered saline (PBS) buffer containing 20 g/L bovine serum, and then were preincubated with 5% powdered skim milk for 30 min to block nonspecific binding. For surface staining of P-gp and MRP1, aliquots of cells were incubated with fluorescein isothiocyanate (FITC)-anti human P-gp, MRP1 (Abcam, Cambridge, UK) or an isotype control antibody (Santa Cruz Biotech, Santa Cruz, CA) for 40 min at 4°C at the recommended dilutions. For detection of α-2, 6 sialylation, cell lysates were incubated with FITC-Sambucus nigra (SNA) lectin (Vector Laboratories, Inc). After repeated centrifugation at 1000 r/min, labeled cells were resuspended in 0.2 ml PBS and were analyzed with FACSCalibur (BD Biosciences, San Jose, CA, USA). Fluorescence intensity was measured by Cell Quest software.

RETRACTED

### Statistical analysis

SPSS17.0 software was used, and each assay was performed at least three times. The data were expressed as mean±SD and Student's t-test was used to determine the significance of differences in multiple comparisons. *P<0.05 was considered to be statistically significant.
